The article "‘Becoming and being online EFL teachers’: Teachers' professional identity in online pedagogy" was published in 2024. Journal: Heliyon.

# ‘Becoming and being online EFL teachers’: Teachers' professional identity in online pedagogy

**DOI:** 10.1016/j.heliyon.2024.e37131

**Published:** 2024-08-30

**Authors:** Mark B. Ulla, William F. Perales, Veronico N. Tarrayo

**Affiliations:** a Walailak University, Thailand; b University of Santo Tomas, Philippines

**Keywords:** English language teaching, Language teacher identity, Online language teaching, Online learning, Teacher professional identity

## Abstract

Teaching online may require teachers to shift to and display a professional identity different from the ones they held in face-to-face classroom teaching. Drawing upon the concept of teacher professional identity (TPI) and employing narrative inquiry as a method, the present study examines how two English as a foreign language (EFL) teachers display their professional identity through reflexivity as they shift experiences of being and becoming online teachers. It also explored how such identity is developed among EFL teachers in Thailand throughout their online teaching experience. The findings underscored how the EFL teachers viewed themselves through reflexivity as beginners as they negotiated their TPI during the sudden transition to online teaching because of the COVID-19 pandemic. Based on the findings, we argue that because TPI is dynamic, the sudden shift to online teaching prompted the teacher-participants to reflect on their experiences and redevelop a professional identity corresponding to online teaching as a new environment. The findings contribute to the literature by highlighting the importance of teachers' reflexivity toward TPI development in online teaching and pedagogy.

## 1 Introduction

The concept of teacher professional identity (TPI) has long been studied in the literature (see Refs. [[1], [2], [3], [4], [5]]), arguing that such an identity is constructed based on teachers' engagements with their profession and their ways of identifying themselves in relation to their roles as schoolteachers. Although the term ‘identity’ reflects the personal projection of a teacher in the classroom and the school, it is shaped by how teachers are influenced by their society, learning networks, and academic orientations. In other words, TPI is “a reflection of the characteristics of the learners and the context of instruction at the level of the classroom, the school, the district, and higher levels of context as these impact on the teacher's aspirations and daily practice” ([4] p. 3) [6]. (2019) describes TPI as the shifting experiences of being, becoming, and belonging as teachers, which can be “understood as multiple, evolving, and constructed in interaction, rather than as stable and somewhat resilient personality traits” (p. 470). In addition, TPI involves the teaching profession, how teachers navigate their profession's nuances and roles in society, and who they are as teachers ([7]).

The article "‘Becoming and being online EFL teachers’: Teachers' professional identity in online pedagogy" was published in 2024. Journal: Heliyon.

Consequently, studying TPI is important because it affects teachers' effectiveness and readiness to adjust to changes in the classroom ([8]). It influences teachers’ attitudes, how they allocate efforts, and whether they pursue chances for professional growth. In other words, it directs them toward views of teaching and learning that are acceptable in their context and culture ([8]).

In language education, while most studies on language teacher identity have been conducted focusing on nonnative English‐speaking teachers' (NNESTs) identity formation ([5,9,10]), language teachers' emotions and strategies ([[11], [12], [13]]), and teacher's agency in developing professional identities ([2,14,15]) [16], (2019) acknowledge that the process of identity development is a challenge that novice language teachers face, which can compromise their dedication to teaching. This challenge faced by language teachers may extend beyond face-to-face classroom teaching, as a number of universities may have embraced the pedagogical innovation of online teaching due to the pandemic. Although most schools may have fully returned to physical classroom teaching, other educational institutions may continue to deliver classes online, shaping a new identity for language teachers. We argue that teaching the language online may require language teachers to shift to and display a professional identity different from the ones they held in face-to-face classroom teaching. Such a shifting of teacher identity may result from teachers' reflexivity and ability to recognize what works best and is not in online pedagogy.

Thus, within the context of online language teaching, TPI also plays an important concept that needs to be understood, especially since teachers' pedagogical experiences and practices are mostly in a physical classroom. However, while TPI has been explored in many language education research, limited studies have explored language teachers’ professional identity in online language teaching [17]. (2022) recognized the lack of studies in the literature, highlighting that “the majority of studies on second/foreign language teacher identity have [so far only] explored the face-to-face environment compared to the technology-assisted language learning (TALL) environment” (p. 396).

Drawing upon the concept of teachers' reflexivity in TPI ([18]) and employing narrative inquiry as a method ([19]), the present study examines how EFL teachers display their professional identity through reflexivity as they shift experiences of being and becoming online teachers. It also explores how such identity is developed among EFL teachers in Thailand throughout their online teaching experience. We define TPI in this article as EFL teachers’ professional perspectives of their online identity, constructed and formed by their constant engagement in their profession, especially in online or remote language teaching.

The article "‘Becoming and being online EFL teachers’: Teachers' professional identity in online pedagogy" was published in 2024. Journal: Heliyon.

### 1.1 Teachers’ reflexivity and TPI

The concept of reflexivity has been used widely in several social science research studies ([18,20]). Although a number of studies have begun to reconceptualize and explore the concept within language and teacher education, many of these studies have used reflexivity as a process that allows for an exploration of institutional language practices, encouraging dialogues and developing awareness of the many uses of a language ([20,21]), including how teachers developed teaching materials in an EFL context ([22]).

[18] (2007) defined reflexivity as “an individual's response to his/her situation, particularly in terms of self-development and the choices available about the future course of his/her life” (p. 75). In other words, reflexivity involves examining and transforming one's self-based on the context and phenomenon that one engages in, especially if such teaching context requires the development of the self, professionally and personally. It may involve “reflecting on one's own multiple, intersecting identities” ([21], p. 583) that enable teachers to acknowledge their language classroom issues ([22]) and address such issues to maximize language teaching and learning [23]. (2014) maintain:

Reflexivity is neither a given nor a static element and, in this regard, involves not only a willingness to recognize and engage with complexities but also necessitates as well as exudes multimodal ways of engaging with representations of social life, particularly those that are unexpected. (pp. 2–3)

Furthermore, reflexivity not only engages teachers in self-reflections of their classroom teaching practices but also allows them to gain an in-depth understanding and learn from their experiences ([24]). We argue that understanding and learning from challenging experiences is essential for developing TPI among teachers.

In the online teaching environment, where EFL teachers may still have tried to understand themselves as online teachers, they may become reflective not only of their teaching practices but also of their professional identity. In this study, the term reflexivity is defined as how EFL teachers perceive their pedagogical practice as they reflect on their experiences of being and becoming online language teachers. We believe that teachers’ reactions to the new online teaching environment, which they may not have experienced before, may require them to question their practices, affecting their professional identity.

The article "‘Becoming and being online EFL teachers’: Teachers' professional identity in online pedagogy" was published in 2024. Journal: Heliyon.

#### 1.1.1 Online language teaching: the Thai context

While several studies have examined English language teacher identity, one area in research that has remained underexplored is language teachers’ professional identity through reflexivity in online language teaching. In the current context of the COVID-19 pandemic, when teaching the English language in most contexts is done remotely or online, it not only alters the pedagogical practices of language teachers ([25]) but also creates an impact on how these teachers perceive and reflect on themselves as online language teachers.

In Thailand, the teaching and learning process in all schools has also been affected by the COVID-19 pandemic. This led to a temporary halt in face-to-face classroom teaching, with some schools transitioning to online and remote methods. Consequently, platforms like Zoom, Microsoft Teams, and Google Classroom may have gained popularity not only for their convenience but also because some schools lack a proper learning management system (LMS). Despite some universities having an established LMS, the sudden onset of the coronavirus caught both the university and its teachers off guard, rendering them unprepared to leverage the existing LMS fully and navigate the challenges in online teaching. Thus, teachers resorted to employing various online platforms to sustain the continuity of the teaching and learning process, which may affect their identities as teachers.

For instance, since online language teaching is a phenomenon that is new to some English language teachers, they may find it challenging, taxing, and overwhelming [25]. (2022) found that “teachers faced issues that challenged their classroom pedagogical practices, doubted their teaching abilities, and questioned the learning outcomes of their students” (p. 1) during the sudden transition to remote and online teaching. Such issues are often linked to language teachers' lack of pedagogical skills to teach online or remotely ([26]). Teachers have had to modify, adapt, and develop teaching materials suitable for online or remote teaching since they may have been designed only for face-to-face classroom teaching. Since teachers’ pedagogical orientation and practice were limited to face-to-face classroom teaching, they may have to upskill themselves to learn online and remote pedagogies. This process requires them to undergo a professional development program and reflexivity that equips them to become remote or online language teachers. Most often, TPI is in question, considering that teachers may have to adapt to the changing educational landscape and may need to develop and demonstrate an identity that is either similar or different from the ones they used to have.

[27] (2021) acknowledged that “online teaching could largely define and (re)shape teachers' identities, sense of agency, and the extent to which they feel belonging to their communities” (p. 3). In their study [27], (2021) examined the identity construction of six teachers as they transitioned from personal to online classes during the COVID-19 pandemic. The researchers found that shifting classes to online influenced various aspects of teachers' identity, particularly teachers’ agency, self-images, emotions, and beliefs.

The article "‘Becoming and being online EFL teachers’: Teachers' professional identity in online pedagogy" was published in 2024. Journal: Heliyon.

While the study by Ref. [27] (2021) may have become an important precedent for the current research, it calls for more studies to understand teachers' reflexivity and professional identity, especially how the transition to online or remote teaching impacts teachers' identity construction. The current study aims to address this gap by shedding new perspectives on teachers' professional identity and reflexivity in online language teaching from university academics in Thailand, a context that is rarely explored and studied. The present study's findings are also expected to have implications for online pedagogy. Specifically, the study seeks answers to the following questions:

1. What perceptions do EFL teachers have in becoming online language teachers?
2. How does their reflexivity in online-teaching experience shape teacher professional identity in online language teaching?

## 2 Method

### 2.1 Narrative inquiry

The current study follows the qualitative research design, employing narrative inquiry as a research method. Narrative inquiry is a research methodology that examines the stories of people's experiences of a phenomenon: “It is the phenomenon studied in inquiry … a way of thinking about the experience” ([28], p. 477). In other words, people who experience the world have stories to tell, and researchers collect, transcribe, describe, and write these stories ([29]) so that others may understand them and be inspired.

Narrative inquiry has become a popular research methodology in educational research because “education is the construction and reconstruction of personal and social stories; teachers and learners are storytellers and characters in their own and others’ stories” ([29], p. 2). Such stories, when shared, are important for understanding how teachers and students live with their everyday experiences that may have shaped their personal or professional perspectives toward teaching and learning.

[28] (2006) emphasized the “three commonplaces: temporality, sociality, and place—which specify dimensions of an inquiry space” (p. 479) in narrative inquiry. These commonplaces are likened to being “in the spirit of checkpoints” (p. 479), providing a framework for the narrative inquiry.

The article "‘Becoming and being online EFL teachers’: Teachers' professional identity in online pedagogy" was published in 2024. Journal: Heliyon.

Moreover [37], (2019) also elaborated further on this three‐dimensional narrative inquiry space, which includes interaction, continuity or temporality, and situation.

Interaction, conceptualized as the link between personal and social factors of experience, involves sharing life experiences through which the storyteller looks inward to their feelings, hopes, and desires, and outward to existential environments. Continuity or temporality involves looking backward to earlier experiences, connecting them with current happenings, and looking forward to the future and experiences that might be implied or anticipated. Situation concerns locations in the storyteller’s geographical spaces that provide added meaning to the stories being told (p. 4).

In the present study, we explore how these three commonplaces of narrative inquiry shaped EFL teachers’ professional identity as they shifted their experiences of being and becoming online teachers at a university in Thailand. We believe that online teaching as a phenomenon would be a good site to explore TPI through a narrative inquiry since teachers are new to this online teaching environment.

### 2.2 Participants

To answer the research questions posed for the study, we drew on the life story narratives of two EFL teachers (pseudonyms were Beth, 34 years old, and Mira, 36 years old) who expressed willingness to participate in the study and share their online teaching experience. Although they were colleagues of the first author teaching in a Thai university, their stories and experiences about professional development and classroom pedagogical practices, including how online teaching shapes teachers' professional identity, were different.

Beth has a Master's degree in Applied Linguistics and has taught general English courses at the university for almost five years. Meanwhile, Mira has a Master's in English and has taught general English courses at the university for four years. Both were new to online teaching and had no experience or training in conducting online or remote teaching.

### 2.3 Data-gathering procedure

Before the study was conducted, approval was sought from the first author's university review board (IRB) for research on human ethics. With its approval (**approval number WUEC-21**–**115**–**01**), the first author invited the participants to be interviewed for the study. A semi-structured interview was conducted face-to-face at the participant's time convenience. Guide questions were prepared, and follow-up questions were asked for clarification. These questions (see Appendix A) explored how EFL teachers display their professional identity as they shift their experiences of being and becoming online teachers and how such identity is developed among EFL teachers in Thailand throughout their online teaching experience.

The article "‘Becoming and being online EFL teachers’: Teachers' professional identity in online pedagogy" was published in 2024. Journal: Heliyon.

The interview, which lasted between 45 and 70 min, was done using the English language, recorded through a mobile phone, and permitted by the participants. Informed consent was obtained from the participants, who were informed about the purpose of the study and promised confidentiality of their stories.

After the interview, the first author transcribed the data and returned the individual transcript to the participants for member checking, acknowledgment, and confirmation ([38]). Participants were told that they could edit and modify the narratives they shared and include only those they wished to be included especially sensitive personal information. Doing member checking, where participants were allowed to modify and edit their narratives, ensured not only apparency but also the trustworthiness and reliability of the data.

When returned, participants were satisfied with their transcripts; hence, they did not change the transcribed data. In addition, after the analysis and write-up of the Findings and Discussion sections of the paper, the researchers provided the participants with a copy of the analysis and discussion to read.

### 2.4 Data analysis

When the transcribed data were returned to the first author after two to five days, the researchers read the transcripts and did the manual coding to develop and generate themes, answering the research questions posed for the study. Manual coding engaged the researchers in the qualitative data, providing them with deeper insights and understanding of the phenomenon under investigation.

Following the three‐dimensional narrative inquiry space ([28]), the researchers introduced, presented, and discussed the participants’ narratives as personal development paths from the past to the present. The original quotations were used to tell the story, which was then analyzed using [30] (2006) six-phase framework for doing a thematic analysis (becoming familiar with the data, generating initial codes, searching for themes, reviewing themes, defining themes, and writing up).

The coded data from the interview were examined closely to highlight the recurring patterns of meaning within the narratives. After this, the researchers categorized the recurring patterns and developed themes that would best describe the life narratives of the participants.

The article "‘Becoming and being online EFL teachers’: Teachers' professional identity in online pedagogy" was published in 2024. Journal: Heliyon.

From the data analysis, the researchers generated six themes written in a sentence format. These themes were: **‘I felt that I was going back to my preservice years,’ ‘Classroom teaching is way different from online teaching,’ ‘Experience is the best teacher,’ ‘I am a beginner, a neophyte,’ ‘It was challenging, but I enjoyed teaching online,’** and **‘I have become a confident online language teacher.’**

## 3 Findings

During the global pandemic, teachers globally faced an unprecedented shift to online teaching, challenging norms and pushing teachers out of their comfort zones. This study explores Beth and Mira's transformative experiences as language teachers navigating online teaching. Beth, an experienced teacher, felt unease entering online teaching, akin to her preservice years. She grappled with student engagement and resource gaps. Mira, a novice to online teaching, faced the shift optimistically but struggled with technology and doubted her effectiveness. Both encountered common issues—student participation and technology challenges—finding innovative solutions. Beth, leveraging experience, relearned online instruction, while Mira, a beginner, became a confident online teacher with supportive peers. Their stories highlight adaptation, resilience, and ongoing professional growth.

## 4 Continuity

### 4.1 Beth: ‘I felt that I was going back to my preservice years.‘

She is used to teaching inside the classroom with her students physically present. Because she had never experienced teaching online, she felt that she was unqualified to teach online. She also thought that she was like a preservice teacher who was still learning how to teach.

When our department chairperson announced that we’re doing online teaching in the middle of the semester, I was scared because I had never tried or studied how to teach online. I was scared that I would not become a good or effective online language teacher. Teaching online was never part of our curriculum in my BA and MA degrees. I have no training, no background about it whatsoever. I felt that I was going back to my preservice years when I had to learn how to teach, manage the classroom, and prepare the lessons. I felt so unqualified.

I remember my first day teaching online when I was anxious about how I would conduct my lesson. Even if I had all my teaching materials ready, especially my PowerPoint, I still felt that there was something that I needed to do to make my online teaching effective. I said effective if my online students have learned something from what I was talking about during our online class. But students were also not used to having an online class. Sometimes, they did not participate in the online activities. When I asked comprehension questions to them, they were silent. Their lack of participation and engagement in my online class made me realize that I should do something about it. I guess I just want my students to learn something from me in the online class. It made me questioned myself and my profession. Teaching online is really new to me.

The article "‘Becoming and being online EFL teachers’: Teachers' professional identity in online pedagogy" was published in 2024. Journal: Heliyon.

## 5 Interaction

### 5.1 ‘Classroom teaching is way different from online teaching.’

Since it was her first time teaching online, she acknowledged some issues she thought she needed to address to make her online class engaging and learning. These issues include the lack of students’ participation and engagement in her online language activities and the lack of teaching and learning resources suitable for the online teaching environment.

The first two weeks into the online teaching, I felt so exhausted because I needed to prepare not only myself but also my teaching materials. I had to search the internet for online teaching resources, activities, and other language teaching materials that I could use to facilitate students' engagement and learning. I had to relearn the skills of teaching and apply those teaching strategies online because classroom teaching is way different from online teaching. When you teach in the classroom, you can physically engage the students in language activities where they can also interact with their classmates, but in online teaching, students are far from each other. And getting them to work on group activities is really a challenge. But every time I logged into my Zoom account to deliver my online teaching, I learned to adapt to its nature. I learned to master some basic skills in using technology and integrating them into my teaching. I think because I also read online teaching articles from journals and participated in online teaching training, seminars, and coaching, I could deliver my online lessons. Teaching online was challenging, but I did it with my colleagues' support. And it was a learning experience. My colleagues were very helpful because we shared some strategies and activities to make our online class as effective as possible.

## 6 Situation

### 6.1 ‘Experience is the best teacher.’

Beth considered her online teaching experience a learning experience. Although she encountered issues in her online teaching, she utilized her existing pedagogical skills and knowledge of the teaching profession to become an effective teacher. Likewise, her online teaching experience made her realize that as a teacher, she still has a lot of things to learn.

I consider online teaching as my greatest professional development activity. I always believe that experience is the best teacher. So, even if I had no prior experience in conducting an online class but because I am a teacher, I used whatever teaching styles and strategies and modified them so I could use them in my online class. My online teaching experience completed my teaching career. Although I still have so many things to learn about conducting online classes, I think I would say that I am now a hybrid teacher who can confidently do face-to-face teaching or online teaching. Online teaching not only makes me realize that I still have a lot of things to learn about improving in my profession, but it also opens my mind to be flexible and adaptive to the changing landscape of education.

The article "‘Becoming and being online EFL teachers’: Teachers' professional identity in online pedagogy" was published in 2024. Journal: Heliyon.

## 7 Continuity

### 7.1 Mira: ‘I am a beginner, a neophyte.’

Although she acknowledged the challenges of online teaching, she was optimistic about it since she thought she would only be working in the comfort of her home. Like Beth, Mira was also new to online teaching and never had any experience or training in conducting online or remote teaching.

We started online teaching in the middle of our third term of the academic year 2019–2020, right? I would say that teaching online was okay; at least we are safe from the virus and can work from home. When I knew that we had to move to online teaching, I felt a bit skeptical because I hadn’t tried doing online classes before. Second, my knowledge of the use of technology wasn’t really that good. I knew that online teaching in our university involved the use of technology, but this technology was not introduced to us. We never had an actual training maybe because it [online teaching] was so sudden. Lastly, I was afraid if I would be able to make it, you know, to become an effective online teacher. At the same time, I was also excited by the thought that I would be able to try to do online teaching. If I would to describe myself as an online language teacher, I would say that I am a beginner, a neophyte. My orientation was on face-to-face teaching and never on online teaching. But I think being an online language teacher during the pandemic was exacting, challenging, and tiring because everything was new. For me, I had to prepare my lessons that could be delivered online. I had to make sure that my language learning activities would work online so that students could participate and learn. But each week of doing online teaching, I realized that I learned from this experience. That’s why I enjoyed teaching online.

## 8 Interaction

### 8.1 ‘It was challenging, but I enjoyed teaching online.’

Like Beth, Mira also expressed that she faced some challenges in online teaching. However, despite these challenges, she was certain to address these issues to continue the teaching and learning process.

The article "‘Becoming and being online EFL teachers’: Teachers' professional identity in online pedagogy" was published in 2024. Journal: Heliyon.

I think the common problems we have in online teaching are students not participating in synchronous group activities, not turning on their cameras, and no interaction from them. But I believe that even if we have the same online teaching issues, we have different groups of students, right? So at the end of the day, you need to reflect on the things you did in your class. Maybe you ask yourself why students were not participating in the group activities and why there was a lack of interaction. For me, my solution to this was putting my students in small groups and letting them have their discussions in the breakout room sessions. I provided them with guide questions and after that they had to report back to the main room with whatever things they discussed in their group. As an online teacher, we need to acknowledge that online teaching is different from classroom teaching and the only way to deal with the issues is to better ourselves. We don’t know much about our profession because we are only confined to teaching in the physical classroom. I guess through this experience we can say that learning new things never ends.

Although Mira considered herself a beginner in online teaching, with no prior training and experience, she nevertheless enjoyed doing it. She learned to adapt to the new normal in education by enhancing her teaching skills. One of the ways she mentioned that helped her address the online teaching issues she encountered was by reflecting on her daily online teaching experience. She acknowledged that she could improve her online teaching skills by engaging in self-reflection, highlighting her teaching practice that needed improvement.

I would say that it was challenging, but I enjoyed teaching online probably because aside from the support from our course coordinators and other colleagues who were also teaching online, I guess because I also assess and reflect on the things I do in my online class. And I like challenges because I learn from them … You know, when you reflect on the things you did, you would be able to identify what went wrong and what went well. I believe this is important because by doing this, you would be able to address those issues to improve your class the next time.

One thing that also helped me get through with online teaching was the support from my colleagues. They say that the more people you travel with, the more exciting it will be. This is I think the best description that I could say regarding my experience in online teaching. My colleagues and I had this group chat, where we exchanged tips and strategies on how to do online teaching. We also shared language teaching and learning materials. So, even if I am new to online teaching, I have a support group that is always there to guide me. Participating in exchanging and sharing teaching resources and strategies is also one of the best professional-development activities. That is why I am glad that I have supportive colleagues.

The article "‘Becoming and being online EFL teachers’: Teachers' professional identity in online pedagogy" was published in 2024. Journal: Heliyon.

## 9 Situation

### 9.1 ‘I have become a confident online language teacher.’

Mira's experience as an online language teacher developed her confidence to teach online. With the support from her colleagues, she faced the challenges positively, allowing her to improve her online teaching skills.

Based on my experience, when you reflect on the things you did in your online language classroom, you will be able to design activities that will surely help you solve those issues you have. Also, when you have a support group that is just so supportive of you, you will be able to face the issues you encountered in online teaching. I would say that I have become a confident online language teacher. Reflective teaching and supportive colleagues boost my confidence. And I also think that even if I have been teaching for almost five years already, I still belong to the new breed of teachers new to online teaching. I take this experience as a memorable one. I considered this the real teacher professional-development activity because I learned a lot from my own experience.

## 10 Discussion

The present study explored the concept of TPI through teachers' reflexivity by employing narrative inquiry to examine how two EFL teachers in Thailand build their professional identity as they shift experiences of being and becoming online teachers. It highlighted that English language teachers’ practices and continuous learning involve the enactment, negotiation, and (trans)formation of their professional identity, which intersperses with their other social identities (e.g., race, gender, ethnicity) and with the varied social situations they encounter.

The findings revealed that reflexivity allows teachers to reflect on their TPI, particularly their personal and professional perspectives of their online identity. Such TPI was constructed and formed by teachers' constant engagement in their profession, especially in the sudden transition to online or remote language teaching. By engaging in reflexivity, teachers acknowledged that conducting online or remote language teaching brought them back to their preservice-teaching years when they were inexperienced teachers who were still learning how to teach. They perceived themselves as neophytes and ‘beginners,’ considering they were not trained to conduct online or remote teaching since their orientation was on face-to-face classroom teaching. They were anxious about how to deliver their online classes and whether they would be effective teachers for their students. They also acknowledged that teaching online or remotely was different from face-to-face teaching since they not only dealt with online pedagogies but also needed to familiarize themselves with some online platforms.

The article "‘Becoming and being online EFL teachers’: Teachers' professional identity in online pedagogy" was published in 2024. Journal: Heliyon.

Although the way they perceived themselves during this emergency transition to online or remote teaching is understandable, it makes the teachers question and doubt their ability and feel threatened and insecure. Previous studies have reported such teachers' perceptions and emotional reactions (see Refs. [[31], [32], [33]]) to a sudden shift to online or remote teaching. The teachers may have felt so stressed about the sudden change of the teaching modality that they thought of themselves as unqualified, considering that they did not have prior online teaching experience. However, these perceptions and attitudes allowed them to form a new identity to cope with the demands of the new educational landscape. In other words, teachers had to contend with challenges in negotiating their identities within the complexities of teacher training, improved educational programs, curricular reforms, professional development training, subject-specific knowledge, and teaching competencies. This implies that certain factors, such as teachers' pedagogical beliefs, positive and negative emotional experiences, and sociocultural contexts, may affect how they perceive themselves as online language teachers, impacting their professional identity.

Thus, teachers became reflective teachers as they engaged in reflective teaching to identify and address issues and maximize students’ learning. In other words, these teachers reflected on their commitment to their profession as they continued to innovate ways to make their online or remote teaching as engaging as possible for their students [34]. (2018) explicated that reflective teaching allows language teachers to examine and identify issues in the language classroom, developing more informed teaching practices and deeply understanding the profession.

The findings also indicated that even if the teachers lacked the knowledge and skills to deliver online or remote language teaching, they became adaptive to the situation. They realized that they still have several things to learn in their teaching profession, especially in the aspect of online or remote teaching. In other words, despite the issues they faced and their lack of skills for online teaching, these teachers did not falter in their commitment to the teaching profession. Instead, they remained committed and enjoyed the new learning experience. They faced and addressed the issues to improve their teaching. This attitude has been described by Ref. [35] (2021) as emotional resilience [35]. (2021) explained that “emotional resilience refers to academics' capacity to bounce back, to thrive amid identity tensions, and to construct integrated professional identities despite emotionally challenging circumstances” (p. 236). The teacher-participants’ emotional resilience can also be argued to be essential in developing their identity in online or remote teaching. For example, while they encountered students’ lack of participation and engagement in group language learning activities as one common issue in their online or remote teaching, they mitigated such an issue by participating in training, seminars, and coaching related to online teaching. They also built a community of support and practice with their colleagues. A study by Ref. [36] (2021b) found that a community of practice played a big role in addressing common issues linked to online teaching. The researchers also reported that teachers who were part of this community of practice not only found a support group and a source of solutions to online teaching problems but also found a learning community where everyone shared their teaching experiences and learned from one another.

The article "‘Becoming and being online EFL teachers’: Teachers' professional identity in online pedagogy" was published in 2024. Journal: Heliyon.

Furthermore, based on the findings, TPI can be regarded as dynamic and is influenced by how the teachers perceive themselves and act in a teaching situation that is new to them. In the context of the COVID-19 pandemic, when there was a sudden shift to online or remote teaching, TPI was developed from the teaching situation needing it. TPI was formed by the acknowledgment of the teachers of the current teaching context and the problems, including their abilities to conduct online or remote teaching. By acknowledging the teaching situation and accepting themselves as unqualified online or remote teachers, they formed their new identity, influenced by their engagement in the teaching practice, professional development activities, and online community. The experience of starting all over again and adapting to the changing landscape of the new normal in teaching assisted in developing their TPI in online or remote teaching. However, it should be noted while such TPI is dynamic, it can be stable at times when teachers are already accustomed to the practice. In the current study, teachers had to modify their attributes to fit the online teaching environment. They may already have formed their TPI in face-to-face classroom teaching, but they had to redevelop their identity because they would face a new teaching environment that they had never experienced before. This was evident in the findings when one of the teachers recognized that online teaching was different from face-to-face teaching. They may have felt anxious about their new teaching experience, but they had to form their identity of being and becoming online or remote language teachers. This finding corroborates what [17] (2022) found about teachers recreating their identity to adapt to the online teaching community [17]. (2022) emphasized that “teachers who were trained to teach in the face-to-face (F2F) environments and had formed particular context-oriented teacher attributes (i.e., relatively stable personality characteristics) have to modify and redevelop new teacher attributes that adapt to the online professional environment” (p. 397).

The article "‘Becoming and being online EFL teachers’: Teachers' professional identity in online pedagogy" was published in 2024. Journal: Heliyon.

Lastly, although the study was conducted during the pandemic, it holds relevance for and contributes to current EFL teaching, teacher identity, and professional development. Emphasizing the importance of teacher reflexivity, it underscores its critical role when adapting to sudden shifts to online or remote teaching. The findings suggest that cultivating teacher reflexivity holds promise for EFL teaching. Thus, reflective practices may not only empower teachers to adjust and forge a new identity aligned with the dynamic demands of the educational landscape, especially during crises like the pandemic, but it also positively impacts the development of a dynamic TPI, enhancing teachers' capacity to navigate and excel in the ever-changing field of education.

Moreover, the study also highlights the dynamic nature of TPI, shaped by teachers' perceptions and actions in new teaching situations, emphasizing that reflective teaching significantly improves practices, fostering a more informed approach. Despite challenges, such as a limited understanding of online or remote language teaching, teachers engaging in reflective practices enhance their professional understanding. In other words, when teachers regularly engage in reflective practices, they may learn new abilities, pinpoint areas for growth, and remain current with best practices. However, teachers must engage in continuous learning and other professional development to succeed in the current educational landscape.

## 11 Conclusion

The present study explored teachers’ reflexivity in online-teaching experience and how it shaped teachers' professional identity. Interview findings revealed that reflexivity allows teachers to reflect on their TPI, particularly their personal and professional perspectives of their online identity, during the sudden transition to online or remote language teaching. These perceptions and attitudes allowed them to form a new identity to cope with the demands of the new educational landscape. The findings also revealed that reflective teaching enables language teachers to develop more informed teaching practices and deepen their understanding of the profession, even if they lack the knowledge and skills to deliver online or remote language teaching. Thus, TPI is dynamic and influenced by how teachers perceive themselves and act in a new teaching situation.

The article "‘Becoming and being online EFL teachers’: Teachers' professional identity in online pedagogy" was published in 2024. Journal: Heliyon.

Furthermore, the findings suggest that TPI, although reflecting individual traits, is developed from teachers’ personal and professional perspectives and their self-reflexivity of their teaching profession, students, and community of practice. It is dynamic and changes based on the needs of the teaching context. As language teachers form their online identity, they not only expand their social network and the sociocultural contexts where they navigate, but they also tend to construct and (trans)form their identities as they interact with new individuals or groups and assume new roles in new communities of practice. In the context of online teaching during the COVID-19 pandemic, such TPI may be constructed and formed as teachers constantly engage, reflect, commit, and practice in their profession. This also suggests that forming TPI in an emergency online teaching requires teachers to acknowledge and recognize the teaching context, including its challenges. By accepting these challenges and adapting to the new teaching environment, teachers may develop an identity that may elicit positive dispositions toward their personal and professional lives.

The study's findings have implications for the teacher education program, particularly for EFL teachers in online pedagogy. First, challenges are part of the teaching experience, especially for EFL teachers new to online pedagogy. These should not be used to determine one's ability to deliver lessons but as a learning experience that could inform one's online pedagogy practice. Second, online pedagogy is different from traditional lecture-discussion pedagogy. Teachers should constantly engage in various professional development programs to cope with the changing needs of teaching and education. Schools should also support their teachers so they may become skillful in online teaching and online pedagogy.

Lastly, although the study reports findings that contribute to the literature on TPI in online teaching and pedagogy, it acknowledges its limitations that future studies may wish to address. For example, the study context was EFL teachers teaching online during the COVID-19 pandemic. Other studies may want to investigate EFL teachers and other teachers in the field to shed new insights on TPI during the pandemic. In addition, a correlational study of teachers’ experience and TPI in online pedagogy can also be interesting to explore.

The article "‘Becoming and being online EFL teachers’: Teachers' professional identity in online pedagogy" was published in 2024. Journal: Heliyon.

## Availability of data and material

Data will be made available on request.

## CRediT authorship contribution statement

**Mark B. Ulla:** Writing – review & editing, Writing – original draft, Conceptualization. **William F. Perales:** Writing – review & editing, Writing – original draft, Methodology. **Veronico N. Tarrayo:** Writing – review & editing, Writing – original draft, Methodology.

## Declaration of competing interest

The authors declare the following financial interests/personal relationships which may be considered as potential competing interests:The first and corresponding author, Dr. Mark Bedoya Ulla, serves as Associate Editor for Heliyon (Education section). If there are other authors, they declare that they have no known competing financial interests or personal relationships that could have appeared to influence the work reported in this paper.

## Appendix A

### Interview Guide Questions

Please give your substantial answer to each question.

1. Can you walk us through your online teaching experience?
2. How do you describe yourself as an online language teacher teaching during the COVID19 pandemic?
3. How do you compare your online teaching and classroom teaching experiences?
4. What do you think were the reasons that affected your teaching practices in online teaching?
5. What challenges have you encountered in your online teaching?
6. Did your challenges change your perspective regarding your teaching practice and your identity as a teacher?
7. How did you address those issues in online teaching?
8. How do you perceive yourself as a language teacher before transitioning to online teaching and during online teaching?
9. How does your online teaching experience shape you as an online language teacher?
10. What have you learned from that online teaching experience?
